# Segmentation of Intensity-Corrupted Medical Images Using Adaptive Weight-Based Hybrid Active Contours

**DOI:** 10.1155/2020/6317415

**Published:** 2020-11-04

**Authors:** Asif Aziz Memon, Shafiullah Soomro, Muhammad Tanseef Shahid, Asad Munir, Asim Niaz, Kwang Nam Choi

**Affiliations:** ^1^School of Computer Science and Engineering, Chung-Ang University, Seoul, Republic of Korea; ^2^Department of Computer Science, Quaid-e-Awam University of Engineering Science and Technology, Shaheed Benazirabad, Pakistan; ^3^Department of Industrial and Information Engineering, Università degli Studi di Udine, 33100 Udine, Italy

## Abstract

Segmentation accuracy is an important criterion for evaluating the performance of segmentation techniques used to extract objects of interest from images, such as the active contour model. However, segmentation accuracy can be affected by image artifacts such as intensity inhomogeneity, which makes it difficult to extract objects with inhomogeneous intensities. To address this issue, this paper proposes a hybrid region-based active contour model for the segmentation of inhomogeneous images. The proposed hybrid energy functional combines local and global intensity functions; an incorporated weight function is parameterized based on local image contrast. The inclusion of this weight function smoothens the contours at different intensity level boundaries, thereby yielding improved segmentation. The weight function suppresses false contour evolution and also regularizes object boundaries. Compared with other state-of-the-art methods, the proposed approach achieves superior results over synthetic and real images. Based on a quantitative analysis over the mini-MIAS and PH^2^ databases, the superiority of the proposed model in terms of segmentation accuracy, as compared with the ground truths, was confirmed. Furthermore, when using the proposed model, the processing time for image segmentation is lower than those when using other methods.

## 1. Introduction

Image segmentation involves segmenting or partitioning a digital image into regions that contain objects of interest; this process is the basis for digital image analyses. Different techniques have been employed for image processing and computer vision in order to segment meaningful regions of interest (ROIs) in images.

Images can be classified as homogeneous or inhomogeneous based on the types of regions they comprise.  Figure 1 presents an example of a homogeneous image with a strongly defined boundary, along with its histogram. Furthermore, Figure 2 depicts an inhomogeneous image along with its histogram, illustrating the inhomogeneity of the image.

Imaging technologies have played a significant role in improving the quality of medical care. By using such techniques, accurate diagnoses for complications in various regions of the body can be realized, such as tumors in the brain, veins, and breasts [1–10]. In medical imaging, tumor boundaries are defined to measure the sizes of the ROIs, thereby providing early cancer diagnoses [11]. However, identifying object details from images obtained via techniques such as magnetic resonance imaging, computerized tomography imaging, and X-ray imaging can be challenging due to the presence of significantly inhomogeneous intensities and blurred object boundaries.

There are different methods to perform image segmentation such as Supervised methods and unsupervised methods. The deep learning relies on the training dataset in deep learning-based image segmentation [12]. The larger and comprehensive datasets are used for better segmentation accuracy and efficiency; however, produce inferior results on small datasets. The level set methods are known as unsupervised methods to perform image segmentation and used preselected parameters, depending on the Region of Interest. The proposed method contributes the unsupervised method and surpasses previous level set methods, in terms of efficiency. Furthermore, the comparison of the proposed method with other state-of-the-art methods and the ground truth performed and shown in the result section.

Active contours, which is an image segmentation technique employing energy minimization for the extraction or separation of ROIs, can be used to overcome these issues. Active contours are computer-generated curves that move under the influence of equal and opposite internal and external forces. Active contour models are categorized into two types: edge-based [13–17] models and region-based [1–10, 18–24] models. Edge-based models employ image gradient-based edge detectors to control contour evolution to the desired object boundaries. These models exhibit inferior performance on images with strong noise, weak edges, and low contrasts. Region-based models offer several advantages over the edge-based models. Region descriptors, commonly employed to control contour evolution, are less sensitive to contour initialization and do not utilize the image gradient. Therefore, images with low contrast and/or weak boundaries can also be segmented successfully.

For instance, the Chan and Vese (C-V) region-based model [2] offers advantages in terms of contour initialization and noise, as compared with edge-based models. However, region-based models tend to perform poorly when the images feature inhomogeneous intensities.

Li improved the C-V model using the local binary fitting (LBF) [3] energy to segment images with intensity inhomogeneity. LBF introduces local minima into energy functionals using local information. However, contour initialization is highly sensitive, which limits its usage in different applications [25]. Chen et al. [7] proposed an improved active contour model for intensity inhomogeneous image segmentation, employing a customized Gaussian kernel bias field estimator to address the inhomogeneity in intensity.

The variational formulation accurately identifies the global energy functional minimum when segmenting images [11, 26–28]. However, the energy functional identifies one segment region at a time, and it was formulated under the assumption that the K-mean characteristic functions are combined linearly and represented as intensity variations [29, 30]. Min et al. [31] proposed a method based on a global division algorithm; this method employed a new global intensity term, which further improved the performance of the C-V model for complex image intensities.

In this study, we formulate a hybrid region-based active contour model with variation level set derivation, using both local and global intensity fitting energy terms. This hybrid model completely eliminates reliance upon the initial contour position and incorporates an adaptive weight function to efficiently segment images with intensity inhomogeneity.  Figure 3 presents the results obtained by applying the proposed method on the homogeneous and inhomogeneous images in Figures 1 and 2, respectively.

The contributions of this study to active contour model-based image segmentation can be summarized as follows:

- A novel hybrid active contour model comprising efficient features of the local region-based and global region-based fitting energies is proposed
- The inclusion of the local region-based ACM statistics ensures that the contour evolution over inhomogeneous regions effectively captures the intensity-corrupted ROI
- The inclusion of the global region-based ACM statistics ensures robust evolution of the contour over homogeneous regions
- The hybrid active contour formulation makes the contour movement independent of the contour initial location, making it less sensitive to the local minima
- The adaptive weight function helps to adapt fitting parameters over object boundaries and contributes to an increase segmentation accuracy

The remainder of the paper is organized as follows.  Section 2 presents a review of standard models and discusses their limitations. The proposed energy model and its level set formulation are described in Section 4.  Section 6 presents the validation of the results of the proposed method for real and synthetic images.  Section 5 discusses various outcomes for the quantitative analysis of the proposed approach, as compared with the ground truths. Finally, Section 6 highlights the conclusions of this research.

## 2. Background Work

### 2.1. Mumford–Shah Model

Mumford and Shah [20] proposed an object functional for image segmentation, defined as follows:

(1) $$\begin{array}{c} E^{\text{MS}}\left(C,u\right)=\lambda \int_{\Omega }{\left|I-u\right|}^{2}dx+v\int_{\Omega \backslash C}{\left|\nabla u\right|}^{2}+\mu \left|C\right|, \end{array}$$

where *Ω* defines an image domain, *I* is the intensity of the original image, *C* is the length of the curve, and *μ* and *v* are positive fixed parameters. The fitting function *u* and the optimal segmenting curve *C* can be obtained via the minimization of the energy functional to approximate *I*.

Thus, the model provides a curve *C*, segmenting the image into several separate ROIs. A fitting function *u* smoothens each subregion and thus estimates the intensity *I* of the original image. However, it is challenging to minimize the energy functional due to the unknown contour *C*. Therefore, various methods have been proposed to modify this energy functional, some of which are discussed below.

### 2.2. Chan–Vese (C-V) Model

The C-V model is a region-based active contour model that overcomes the shortcomings of the Mumford–Shah model [20] by using a simple assumption that the image intensities in each ROI are constant. The energy functional in the C-V model is expressed as

(2) $$\begin{array}{c} E^{\text{CV}}\left(C,e_{1},e_{2}\right)=\lambda_{1}\int_{\Omega }{\left|I\left(x\right)-e_{1}\right|}^{2}\;H_{\varepsilon }\left(\phi \;\left(x\right)\right)dx+\lambda_{2}\int_{\Omega }{\left|I\left(x\right)-e_{2}\right|}^{2}\;\left(1-H_{\varepsilon }\left(\phi \;\left(x\right)\right)\right)dx+\mu .\text{Length}\left(C\right)+v.\left|C\right|, \end{array}$$

where *I*(*x*) represents the image being analyzed, and the global fitting energies *e*_1_ and *e*_2_ are the image intensities inside and outside the contour *C*, respectively. *λ*_1_,  *λ*_2_, *μ*, and *v* are positive parameters, and area (*C*) is the Heaviside function. On minimizing equation (2) with respect to *e*_1_, *e*_2_, and *ϕ* using the gradient descent [28], we obtain

(3) $$\begin{array}{c} e_{1}=\frac{\int_{\Omega }I\left(x\right)H_{\varepsilon }\left(\phi \left(x\right)\right)dx}{\int_{\Omega }H_{\varepsilon }\left(\phi \left(x\right)\right)dx}, \end{array}$$

(4) $$\begin{array}{c} e_{2}=\frac{\int_{\Omega }I\left(x\right)\left(1-H_{\varepsilon }\left(\phi \left(x\right)\right)\right)dx}{\int_{\Omega }\left(1-H_{\varepsilon }\left(\phi \left(x\right)\right)\right)dx}, \end{array}$$

(5) $$\begin{array}{c} \frac{\partial \phi }{\partial t}=\left(-\lambda_{1}{\left(I-e_{1}\right)}^{2}\right)+\lambda_{2}{\left(I-e_{2}\right)}^{2}+\mu div\left(\frac{\nabla \phi }{\left|\nabla \phi \right|}-v\right)\delta_{\varepsilon }\left(\phi \right), \end{array}$$

where *H* is the Heaviside function, with the Dirac delta function *σ*, and *ϵ* is a constant that controls the Dirac delta smoothness and the width in *H*. Approximations for the Dirac and Heaviside functions are as follows:

(6) $$\begin{array}{c} H_{\epsilon }\left(\phi \right)=\frac{1}{2}\left(1+\frac{2}{\pi }\arctan\left(\frac{\phi }{\epsilon }\right)\right), \end{array}$$

(7) $$\begin{array}{c} \delta_{\epsilon }\left(\phi \right)=\frac{\epsilon }{\pi \left(\phi^{2}+\epsilon^{2}\right)}. \end{array}$$

In case of inhomogeneous images, the global fitting energy terms fail to provide sufficient statistics to the C-V model, resulting in unsatisfactory segmentation over inhomogeneous regions. Although the C-V model shows satisfactory performance for homogeneous images, its limitation for inhomogeneous images makes it less preferred.

### 2.3. Local Binary Fitting Model

The LBF model segments images with intensity-corrupted regions and overcomes the limitations of the C-V model. The energy fitting model in LBF is defined as

(8) $$\begin{array}{c} E_{\text{LBF}}\left(C,h_{1},h_{2}\right)=\lambda_{1}\int_{\Omega }G_{\sigma }\left(x-y\right){\left(I\left(y\right)-h_{1}\left(x\right)\right)}^{2}.H_{\epsilon }\left(\phi \left(y\right)\right)dy+\lambda_{2}\int_{\Omega }G_{\sigma }\left(x-y\right){\left(I\left(y\right)-h_{2}\left(x\right)\right)}^{2}.\left(1-H_{\epsilon }\left(\phi \left(y\right)\right)\right)dy, \end{array}$$

where *G*_*σ*_ represents the Gaussian kernel function with the standard deviation *σ*. The LBF energy functional can be represented in a level set formulation by minimizing equation (6) with respect to the local intensity means inside and outside the regions, termed as *h*_1_ and *h*_2_, respectively. These can be defined using the gradient descent as follows [28]:

(9) $$\begin{array}{c} h_{1}\left(x\right)=\frac{G_{\sigma }*\left[H_{\epsilon }\;\left(\phi \left(x\right)\right)\;I\left(x\right)\right]}{G_{\sigma }*H_{\epsilon }\left(\phi \left(x\right)\right)},\\ h_{2}\left(x\right)=\frac{G_{\sigma }*\left[\left(1-H_{\epsilon }\;\left(\phi \left(x\right)\right)\right)\;I\left(x\right)\right]}{G_{\sigma }*\left(1-H_{\epsilon }\left(\phi \left(x\right)\right)\right)}. \end{array}$$

LBF can segment inhomogeneous images using the local statistical information in a timeframe to decide the direction of contour evolution. Although LBF outperforms the C-V model in inhomogeneous image segmentation, it misses obscured boundaries in some inhomogeneous images. This is because the local intensity means statistics are insufficient to provide accurate segmentation results in every scenario.

Figure 4 shows an example image with a blue rectangle and red outline, representing the initial contour and the evolving segmentation curve, respectively. The pixel *p*_1_ is on the less inhomogeneous region; thus, the contour stops evolving at this level. The local intensity means *h*_1_ and *h*_2_ are unable to capture regions with increased inhomogeneity levels. Therefore, pixels *p*_2_ and *p*_3_ are determined at uncertain positions by the LBF model.

### 2.4. Min Et al.'s Model

The model proposed by Min et al. in [31] includes an effective global term to help segment ROIs with complicated intensity in noisy images, which the C-V model struggles to segment accurately. The global term is an energy functional based on a global division algorithm that develops a new ROI-based term to accurately segment objects with large intensity differences and significant noise. This global energy functional is defined as

(10) $$\begin{array}{c} E_{\mathrm{Min}}\left(\phi ,e_{1},e_{2},g_{11},g_{12},g_{21},{\text{g}}_{22}\right)=\int_{\Omega }H\left(I\left(x\right)-e_{1}\right)\;{\left(I\left(x\right)-g_{11}\right)}^{2}\;H_{\epsilon }\;\left(\phi \left(x\right)\right)dx+\int_{\Omega }\left(1-H\left(I\left(x\right)-e_{1}\right)\right)\;{\left(I\left(x\right)-g_{12}\right)}^{2}\;H_{\epsilon }\;\left(\phi \left(x\right)\right)dx+\int_{\Omega }H\left(I\left(x\right)-e_{2}\right)\;{\left(I\left(x\right)-g_{21}\right)}^{2}\left(1-H_{\epsilon }\;\left(\phi \left(x\right)\right)\right)dx+\int_{\Omega }\left(1-H\left(I\left(x\right)-e_{2}\right)\right)\;{\left(I\left(x\right)-g_{22}\right)}^{2}\left(1-H_{\epsilon }\;\left(\phi \left(x\right)\right)\right)dx, \end{array}$$

where *H*(*I*(*x*) − *e*_1_) and *H*(*I*(*x*) − *e*_2_) are the intensity magnitudes. This method has the advantage of simultaneous calculation of the intensity means from the regions inside and outside the object. On minimizing equation (10) with respect to *g*_11_, *g*_12_, *g*_21_, and *g*_22_ the steepest gradient descent, we obtain

(11) $$\begin{array}{c} g_{11}=\frac{\int_{\Omega }\left(H\left(I\left(x\right)-e_{1}\right)\right)I\left(x\right)H_{\epsilon }\left(\phi \left(x\right)\right)dx}{\int_{\Omega }\left(H\left(I\left(x\right)-e_{1}\right)\right)H_{\epsilon }\left(\phi \left(x\right)\right)dx},\\ g_{12}=\frac{\int_{\Omega }\left(1-H\left(I\left(x\right)-e_{1}\right)\right)I\left(x\right)H_{\epsilon }\left(\phi \left(x\right)\right)dx}{\int_{\Omega }\left(1-H\left(I\left(x\right)-e_{1}\right)\right)H_{\epsilon }\left(\phi \left(x\right)\right)dx},\\ g_{21}=\frac{\int_{\Omega }\left(H\left(I\left(x\right)-e_{2}\right)\right)I\left(x\right)\left(1-H_{\epsilon }\left(\phi \left(x\right)\right)\right)dx}{\int_{\Omega }\left(H\left(I\left(x\right)-e_{2}\right)\right)\left(1-H_{\epsilon }\left(\phi \left(x\right)\right)\right)dx},\\ g_{22}=\frac{\int_{\Omega }\left(1-H\left(I\left(x\right)-e_{2}\right)\right)I\left(x\right)\left(1-H_{\epsilon }\left(\phi \left(x\right)\right)\right)dx}{\int_{\Omega }\left(1-H\left(I\left(x\right)-e_{2}\right)\right)\left(1-H_{\epsilon }\left(\phi \left(x\right)\right)\right)dx}, \end{array}$$

where *g*_11_ and *g*_12_ are the larger and smaller mean intensity values inside the contour, respectively. *g*_21_ and *g*_22_ are the larger and smaller intensities outside the contour, respectively. Min et al.'s model reduces the probability of errors during segmentation in the presence of larger intensity differences, as compared with the C-V model.

Figure 5 presents the segmentation results for a complex image obtained using the C-V model and Min et al.'s model. The C-V method yields inferior segmentation due to the noise dots forming individual ROIs, whereas Min et al.'s model yields superior segmentation accuracy.

## 3. Proposed Model

The proposed energy functional is formulated by combining gainful features of both the local and global fitting models. An adaptive weight function is appended with the hybrid energy functional to parameterize weight coefficients for images with different levels of intensity corruption. The global fitting part of the proposed model is termed as the global fitting energy support function (*F*_GFES_), and it is defined as

(12) $$\begin{array}{c} F_{\text{GFES}}=p\left[\frac{h_{1}+h_{2}}{\alpha }\right]\left(\text{Avg}\left(I_{T}\right)\right)-p\left[\frac{h_{1}+h_{2}}{\alpha }\right]\left(\text{Avg}\left(I_{T}\right)\right).\left(I_{T}\right) \end{array}$$

where *Avg*(*I*_*T*_) is the average intensity of the image under analysis and reflects the global contrast for the image, *p* ∈ [0, 1], where *p* denotes positive fixed parameters. The image intensity is defined as

(13) $$\begin{array}{c} I_{T}=\frac{1}{I_{g}}\;\left(I_{\max}-I_{\min}\right), \end{array}$$

where *T* defines the local window size, *I*_max_ is the maximum intensity level, and *I*_min_ is the minimum intensity level within the local window. The overall image intensity level is represented by *I*_*g*_, and it is typically 255 for grayscale images. *I*_*T*_ ∈ [0, 1] reflects the rate of intensity changes in a local ROI. It is smaller for smooth ROIs and larger for ROIs near the object boundaries. Thus, the proposed energy functional, incorporating both global and local fitting energy terms as well as the adaptive weight function, is expressed as

(14) $$\begin{array}{c} E_{\text{LGEF}}\left(u,C\right)=\left.\lambda_{1}\int_{\Omega }\;G_{\sigma }\left(x-y\right)\right|I\left(y\right)-h_{1}{\left|{}^{2}\;H_{\epsilon }\left(\phi \left(y\right)\right)dy+\lambda_{2}\int_{\Omega }\;G_{\sigma }\left(x-y\right).{\left|I\left(y\right)-h_{2}\right|}^{2}\left(1-H_{\epsilon }\left(\phi \left(y\right)\right)\right)dy-F_{\text{GFES}}\left(\lambda_{1}\int_{\Omega }\;G_{\sigma }\left(x-y\right)\right|I\left(y\right)-h_{1}\right|}^{2}\;H_{\epsilon }\left(\phi \left(y\right)\right)dy-\lambda_{2}\int_{\Omega }\;G_{\sigma }\left(x-y\right).{\left|I\left(y\right)-h_{2}\right|}^{2}\;\left(1-H_{\epsilon }\left(\phi \left(y\right)\right)\right)dy-\int_{\Omega }\;H\left(I\left(x\right)-e_{1}\right){\left(I\left(x\right)-g_{11}\right)}^{2}\;H_{\epsilon }\left(\phi \left(x\right)\right)dx-\int_{\Omega }\;\left(1-H\left(I\left(x\right)-e_{1}\right)\right){\left(I\left(x\right)-g_{12}\right)}^{2}\;H_{\epsilon }\left(\phi \left(x\right)\right)dx-\int_{\Omega }\;\left(1-H\left(I\left(x\right)-e_{2}\right)\right){\left(I\left(x\right)-g_{21}\right)}^{2}\left(1-H_{\epsilon }\left(\phi \left(x\right)\right)\right)\;dx-\int_{\Omega }\;\left(1-H\left(I\left(x\right)-e_{2}\right)\right){\left(I\left(x\right)-g_{22}\right)}^{2}\;\left(1-H_{\epsilon }\left(\phi \left(x\right)\right)\right)dx-v\left(\int_{\Omega }\;\left|\nabla H\phi \left(x\right)\right|dx\right.+\mu \frac{1}{2}{\left(\left|\nabla \phi \left(x\right)\right|-1\right)}^{2}dx. \end{array}$$

The primary objective is to set the adaptive weight parameter for the global fitting energy term dynamically. The value of the weight parameter ranges from 0 to 1, depending on the inhomogeneity level of the image. Small values account for low levels of inhomogeneity, whereas high values account for high levels of inhomogeneity in the image. Therefore, in the proposed method, the global fitting energy weight function is increased to ensure accurate active contour evolution for inhomogeneous images.

Thus, minimizing *E*_LGEF_ with respect to *ϕ* by utilizing the steepest gradient descent method, we obtain

(15) $$\begin{array}{c} \frac{\partial \phi }{\partial t}=\delta_{\epsilon }\left(\phi \right)\left({\left.\left(1-F_{\text{GFES}}\right)\left(-\lambda_{2}\int_{\Omega }\;G_{\sigma }\left(x-y\right)\;|\;I\left(y\right)\right.-h_{1}\left(x\right)\right|}^{2}dy+\lambda_{2}\int_{\Omega }\;G_{\sigma }\left(x-y\right)\left|{\left.I\left(y\right)-h_{2}\left(x\right)\right|}^{2}dy\right)+F_{\text{GFES}}\left(-\lambda_{1}H_{\epsilon }\left(1-e_{1}\right){\left(1-g_{11}\right)}^{2}\right.-\lambda_{1}\left(1-H_{\epsilon }\left(1-e\right)\right){\left(1-g_{12}\right)}^{2}+\lambda_{2}H_{\epsilon }\left(1-e_{2}\right){\left(1-g_{21}\right)}^{2}+\lambda_{2}\left(\left(1-H_{\epsilon }\left(1-e_{2}\right)\right){\left(1-g_{22}\right)}^{2}\right)\right.+v\delta_{\epsilon }\left(\phi \right)\mathrm{div}\left(\frac{\nabla \phi }{\left|\nabla \phi \right|}\right)+\mu \left(\nabla^{2}\phi -\mathrm{div}\;\left(\frac{\nabla \phi }{\left|\nabla \phi \right|}\right)\right). \end{array}$$

The proposed formulation eliminates computationally expensive reinitialization, by using the penalizing energy term from [1]. The initial level set function in the proposed method is defined as

(16) $$\begin{array}{c} \phi \left(x,t=0\right)=\left\{\begin{array}{cc} -\rho & x\;\epsilon \;\Omega_{0}-\partial \Omega_{0}\\ 0 & x\;\epsilon \;\Omega_{0}\\ \rho & x\;\epsilon \;\Omega -\Omega_{0} \end{array}\right., \end{array}$$

where *ρ* > 0 is a constant. Finally, the algorithm of the proposed method is as follows.

1. Initialize the proposed level set function *ϕ*(*x*) using *ϕ*_0_ from equation (16)
2. Calculate *h*_1_ and *h*_2_ using equation (9).
3. Calculate *e*_1_, *e*_2_, *g*_11_, *g*_12_, *g*_21_, and *g*_22_ using equations (3), (4), and (11), respectively
4. Add the weight function using equation (12).
5. Compute the partial differential equation for *ϕ*(*x*) with equation (15).
6. Return to step (2) until convergence

## 4. Results

The proposed method is tested using synthetic and real images, and it is quantitatively analyzed on two different datasets: mini-MIAS [32] and PH^2^ [33]. All experiments were performed using MATLAB 2018, on a Windows 10 operating system with a 3.40 GHz Intel Core-i7 processor and 16 GB RAM.  Table 1 lists the parameters used in the experiments, including the default parameters of compared methods, for segmenting inhomogeneous intensity images using the proposed method.

Figure 6 presents the results of the inhomogeneous intensity image segmentation achieved using the LBF and proposed methods, for an original image with an initial contour. It can be seen that, unlike the LBF model, the proposed method segmented the image accurately. Furthermore, Figure 7 shows the segmentation results for four medical images with inhomogeneous intensities. From the results, it is evident that the proposed method achieves superior segmentation accuracy and is also time-efficient during the medical image segmentation.

Figure 8 shows the real medical images used to validate the accuracy and time efficiency of the proposed method. The proposed method fitted the contour smoothly within a minimum amount to time.  Figure 9 shows the segmentation results for the synthetic images. Our method achieves improved segmentation accuracy on the synthetic images. The second column in Figure 9 shows the results of the proposed method after five iterations, and the third column shows the results of the proposed method.

Figure 10 compares the segmentation results for medical images obtained using the LBF, Min et al.'s, and proposed methods. The LBF contours tend to be close to the boundaries, with clear segmentation noise in the images; images processed using Min et al.'s method are inaccurately segmented for a few ROIs with weak boundaries. On the contrary, the proposed method yields good segmentation for all images with different levels of inhomogeneous intensities.

Figure 11 compares the segmentation results of different synthetic images obtained using LBF, Min et al.'s, and proposed methods. The images processed using LBF are inefficiently segmented when the intensity levels change, whereas the images processed using Min et al.'s method exhibit inaccurate segmentation on ROI boundaries where the intensity levels change smoothly. However, all the object boundaries are accurately segmented when using the proposed method.

Figure 12 presents synthetic images with different intensities segmented using C-V, LBF, Min et al.'s, FRAGL [34], and proposed methods. The CPU times for the C-V and LBF models were longer than those for the other models. This is because these methods employ convolution, which requires additional time for convergence. Segmentation using Min et al.'s model was generally smooth for the homogeneous intensity images. Results of the FRAGL model were segmented to the object boundary, although the contour moved smoothly to the object; however, these results were not accurate at the boundary. The proposed method yielded more accurate segmentation than the other methods, requiring minimum time and lesser iterations to converge the contours to object boundaries.

Figure 13 compares real-life images with different inhomogeneous intensity levels, for C-V, LBF, Min et al.'s, FRAGL [34], and proposed methods. The FRAGL model achieved improved segmentation accuracy with minimum CPU time and lower number of iterations; however, the proposed method was more efficient. Thus, objects within the images were segmented according to the differences in their intensities.

## 5. Quantitative Comparison

We compared the results of the proposed method against the ground truths and other state-of-the-art methods.

The mini-MIAS database is an open source dataset for breast tumor detection.  Figure 14 shows example mammograms from the mini-MIAS database used for quantitative results, and it investigates advantages of the proposed method. We compared the segmentation methods using an accuracy metric defined as

(17) $$\begin{array}{c} \text{Accuracy}=\frac{\text{TP}+\text{TN}}{\text{TP}+\text{TN}+\text{FP}+\text{FN}}, \end{array}$$

where TP denotes the true positive segmented regions, TN denotes the true negative unsegmented regions, FP denotes false positives, and FN denotes false negative, i.e., the undetected tumor regions.  Table 2 presents the statistics of the segmentation accuracy of Figure 14 as compared with other methods, based on the ground truth.  Figure 15 indicates that the segmentation accuracy of the proposed method is significantly higher than that of the previous methods.

The PH^2^ database [33] was developed to encourage comparative studies for classification algorithms and the segmentation of dermoscopic images. We compared the results of the proposed method with other state-of-the-art methods using the metric for segmentation accuracy defined in equation (17).  Figure 16 shows the segmentation results for example images from the PH^2^ database using the proposed method and comparisons with the ground truth. The green contour indicates the ground truth, whereas the red contour indicates the segmentation via the proposed method. From the figure, it is evident that the proposed method exhibits suitable accuracy for the segmentation of the example images.  Table 3 presents a comparison of the accuracy, number of iterations, and the CPU time of the proposed method on the PH^2^ database [33] with other state-of-the-art methods. The overall accuracy of the segmentation results proves that the proposed method offers superior performance. Moreover, compared with other methods, the number of iterations and the CPU times of the proposed method proves the time efficiency of our model.

## 6. Conclusion

We propose a novel hybrid active contour model integrating local and global fitted energy terms, with an adaptive weight function. The weight function uses global contrast statistical information to adapt the weight parameters dynamically. The proposed method improves image segmentation accuracy for regions with homogeneous and inhomogeneous intensities, and its contour stability and smoothness around accurate object boundaries are confirmed using both local and global statistics. Furthermore, the inclusion of the Gaussian kernel eliminates the need for a reinitialization time, making the proposed model independent of the initial contour positions. Compared to other state-of-the-art models, the proposed method offers superior performance for real and synthetic images with various inhomogeneous intensity levels, as well as significant improvements in terms of segmentation accuracy and processing time efficiency. Furthermore, quantitative comparisons proved the superiority of the proposed approach.

## Figures and Tables

**Figure 1:** Example of a homogeneous image and its histogram.

**Figure 2:** Example of an inhomogeneous image and its histogram.

**Figure 3:** Results of the proposed method over the homogeneous and inhomogeneous images.

**Figure 4:** Image with local and global forces.

**Figure 5:** Segmentation results for a complex image using (a) C-V model and (b) Min et al.'s model.

**Figure 6:** Original image with an initial contour on the left, result of the LBF model in the middle, and result of the proposed method on the right.

**Figure 7:** Real medical images: column 1=original images with initial contours, column 2=proposed method after ten iterations, and column 3=results of the proposed method.

**Figure 8:** Real medical images: column 1=original images with initial contours, column 2=proposed method after ten iterations, and column 3=results of the proposed method.

**Figure 9:** Synthetic images: column 1=original images with initial contours, column 2=proposed method after five iterations, and column 3=results of the proposed method.

**Figure 10:** Real medical images with different inhomogeneous intensity levels: column 1=original images with initial contour, column 2=LBF, column 3=Min et al.'s model, and column 4=proposed method.

**Figure 11:** Synthetic images with various inhomogeneous intensity levels: column 1=original images with initial contour, column 2=LBF, column 3=Min et al.'s model, and column 4=proposed method.

**Figure 12:** Synthetic images with different inhomogeneous intensity levels: column 1=original images with initial contour, column 2=ground truth, column 3=C-V, column 4=LBF, column 5=Min et al.'s model, column 6=FRAGL model, and column 7=proposed method.

**Figure 13:** Real images with different inhomogeneous intensity levels: column 1=original images with initial contour, column 2=ground truth, column 3=C-V, column 4=LBF, column 5=Min et al.'s model, column 6=FRAGL model, and column 7=proposed method.

**Figure 14:** Typical mammogram images: column 1=original images with initial contour, column 2=ground truth, column 3=C-V, column 4=LBF, column 5=Min et al.'s model, column 6=FRAGL model, column 7=Asim et al.'s [28], and column 8=proposed method.

**Figure 15:** Segmentation accuracy graph for the mini-MIAS database.

**Figure 16:** Results of the proposed method for dermoscopic images in the PH^2^ database: green contours represent the ground truth, and red contours denote the results.

**Table 1:** Default parameters.

Parameter/symbol	Values					
	C-V	LBF	Min et al.'s	FRAGL	Asim et al.'s	Proposed
Gaussian kernel *σ*	3.0	3.0	3.0	2.0	2.5	5.0
Initial level set *λ*_1_ = *λ*_2_	1	1	1	1	2	1
Time step *∆t*	0.1	0.1	0.1	0.1	0.01	0.1
*μ*	—	1.0	1.0	1.0	—	1.0
Length term *v*	0.1	0.001 × 255 × 255	0.001 × 255 × 255	0.001 × 255 × 255	0.00001 × 255 × 255	0.01 × 255 × 255
Weight *ω*	—	—	0.01	—	[0,1]	[0, 1]

**Table 2:** Segmentation accuracy of mammogram images.

	Methods					
	C-V model	LBF	Min et al.'s model	FRAGL model	Asim et al.'s	Proposed method
Figure 14, row 1	0.8458	0.9228	0.9325	0.9585	0.9598	0.9628
Figure 14, row 2	0.5568	0.8932	0.9125	0.9238	0.9448	0.9643
Figure 14, row 3	0.6856	0.8254	0.9283	0.9478	0.9518	0.9764
Figure 14, row 4	0.5793	0.8395	0.6523	0.9539	0.9582	0.9718

**Table 3:** Comparison of the proposed method with other methods over the PH^2^ database [33].

Method	Accuracy	Iterations	CPU time (s)
C-V Model [2]	87.7	20	4.622
LBF [3]	86.5	50	12.577
Min et al.'s Model [31]	94.9	33	18.122
FRAGL Model [34]	95.5	28	16.214
Asim et al.'s [28]	95.8	26	15.128
Proposed method	97.6	22	12.245

## Data Availability

We have used different images (synthetic and real) publicly available on the internet. In comparison, the other databases are used for quantitative comparison are listed below with references. (1) The mini-MIAS database, to encourage comparative studies for classification algorithms and the segmentation of mammogram images, is publicly available that can be accessed at http://peipa.essex.ac.uk/info/mias.html. (2) The PH2 database, to encourage comparative studies for classification algorithms and the segmentation of dermoscopic images, is included within the article doi:10.1109/EMBC.2013.6610779.
